# Effects of Out-of-Hospital Continuous Nursing on Postoperative Breast Cancer Patients by Medical Big Data

**DOI:** 10.1155/2022/9506915

**Published:** 2022-01-06

**Authors:** Peijuan He, Bing Zhang, Songna Shen

**Affiliations:** Breast Center, Women and Children's Hospital of Ningbo City, Ningbo 315012, China

## Abstract

This study aimed to explore the application value of the intelligent medical communication system based on the Apriori algorithm and cloud follow-up platform in out-of-hospital continuous nursing of breast cancer patients. In this study, the Apriori algorithm is optimized by Amazon Web Services (AWS) and graphics processing unit (GPU) to improve its data mining speed. At the same time, a cloud follow-up platform-based intelligent mobile medical communication system is established, which includes the log-in, my workstation, patient records, follow-up center, satisfaction management, propaganda and education center, SMS platform, and appointment management module. The subjects are divided into the control group (routine telephone follow-up, 163) and the intervention group (continuous nursing intervention, 216) according to different nursing methods. The cloud follow-up platform-based intelligent medical communication system is used to analyze patients' compliance, quality of life before and after nursing, function limitation of affected limb, and nursing satisfaction under different nursing methods. The running time of Apriori algorithm is proportional to the data amount and inversely proportional to the number of nodes in the cluster. Compared with the control group, there are statistical differences in the proportion of complete compliance data, the proportion of poor compliance data, and the proportion of total compliance in the intervention group (*P* < 0.05). After the intervention, the scores of the quality of life in the two groups are statistically different from those before treatment (*P* < 0.05), and the scores of the quality of life in the intervention group were higher than those in the control group (*P* < 0.05). The proportion of patients with limited and severely limited functional activity of the affected limb in the intervention group is significantly lower than that in the control group (*P* < 0.05). The satisfaction rate of postoperative nursing in the intervention group is significantly higher than that in the control group (*P* < 0.001), and the proportion of basically satisfied and dissatisfied patients in the control group was higher than that in the intervention group (*P* < 0.05).

## 1. Introduction

Breast cancer is one of the most common malignant tumors in women, and the incidence of breast cancer worldwide is as high as about 20% among female malignant tumors [1]. There are about 27.89 new cases of breast cancer in China every year, accounting for 7.82% of female deaths from cancer [2]. At present, breast cancer is mainly treated by surgery, and the 5-year survival rate of patients is about 70% [3], but patients will have postoperative complications such as lymphedema and upper limb dysfunction [4], which seriously affects the postoperative quality of life of patients. Continuous nursing is the extension of medical care to the community, which can achieve the prevention of complications and coordinated care [5]. Studies have pointed out that continuous nursing intervention for postoperative patients with breast cancer can significantly reduce the occurrence of postoperative lymphedema and related symptoms [6]. Continuous nursing intervention can also significantly improve patients' physical, psychological, social, and behavioral health after surgery [7, 8]. The commonly used continuous nursing methods in China are mainly telephone follow-up and home visit. However, due to the limitation of time and space, traditional methods are prone to lost follow-up and have poor nursing effect and lack personalized continuous nursing care for patients [9].

In recent years, with the continuous development of medical service information, intelligent medical treatment has obvious advantages in improving hospital service level and doctor work efficiency [10]. Mobile health (mHealth) refers to a new intelligent medical way that provides medical services and related information through mobile communication tools such as computers, mobile phones, and satellite communications [11]. The mobile medical information platform is convenient, intelligent, and personalized through the mode of “medical + Internet” [12], which can effectively and timely feedback patient care-related information. However, the current mobile medical platform lacks a scientific guidance system, resulting in unsatisfactory intervention effect [13]. Electronic medical record (EMR) is a synthetic system used to electronically record and store clinical diagnosis and treatment records and intervention information of outpatients, emergency patients, and inpatients by medical institutions. In recent years, mobile medical applications based on the cloud platforms have made significant breakthroughs in disease prevention, disease monitoring, and prognosis evaluation [14]. Nevertheless, there lacks an evidence to prove their usability, effectiveness, and safety, and the user viscosity of mobile medical products is poor between different studies [15], which brings potential hazards to patients.

To sum up, the continuous nursing intervention has obvious application value in postoperative nursing care of breast cancer. Mobile medical equipment can overcome the limitations of continuous nursing intervention in time and space, but it still has some shortcomings, such as poor user viscosity and differences in evaluation results, which need to be further optimized. In this study, an intelligent follow-up medical communication system is established based on medical big data and cloud follow-up platform in the Yihui system of Hangzhou Jianhai Technology Co., Ltd, and it is analyzed from the aspects of medical big data mining method and continuous nursing system design, which expected to provide a reference for the evaluation of postoperative intervention effects under big data.

## 2. Materials and Methods

### 2.1. Overall Design of Intelligent Follow-Up Medical System Based on the Cloud Platform

The intelligent medical system based on the cloud platform mainly includes three modules: cloud follow-up system terminal, Web server, and database, involving four layers: client layer, communication network layer, business logic layer, and data layer. The data layer is the bottom layer of the whole system, mainly including the functions of data organization, storage, and transmission. The business logic layer is mainly composed of Java server and REST interface, and the data are managed manually through the Web server, which provides a guarantee for the cloud follow-up system terminal to access the server. The communication network layer mainly expounds the access mode of the cloud follow-up system terminal. The cloud follow-up system terminal mainly interacts with users. The system terminal is connected to the computer so that the user can dial up directly with headphones, send text messages, or send two-dimensional codes to fill in forms to ensure the timeliness and accuracy of data.  Figure 1 shows the overall framework of the intelligent follow-up medical communication system based on the cloud platform of the HUI system of Hangzhou Jianhai Technology Co., Ltd.  Figure 1 shows the overall framework of intelligent follow-up medical system based on the cloud platform.

### 2.2. Medical Big Data Mining Based on the Apriori Algorithm

Medical big data system mainly includes data source, data collection, data storage, data analysis, data service, and data application [16, 17]. Data mining is the process of effectively classifying and extracting different data types in medical institutions through a data mining model. Due to the characteristics of high latitude, medical big data have the phenomenon of overfitting in the data mining process [18]. The Apriori algorithm is a commonly used mining method at present. Its main idea is to find candidate frequent item sets based on a two-stage frequency set recursive algorithm, which has the characteristics of simple operation, easy operation, and low data requirements [19].

Assume *Z* is the item set in all transactions, and for the given minimum support Minsup, if the proportion of item set *Z* in all transactions is higher than or equal to Minsup, item set *Z* is called frequent item set. Frequent item set *Z* must meet the condition of (1). *Z*.con indicates the number of transactions containing item set *Z*, and *n* is the total number of transactions.

(1) $$\begin{array}{c} \frac{Z.\text{con}}{n}\geq \min\;\sup. \end{array}$$

If item sets *A* and *B* are subsets of *M*, *A* and *B* meet *A*∩*B* ≠ ∅, and the proportion of transactions containing *A* ∪ *B* in transaction set *R* to all transactions is called the support degree of association rules *A*⟶*B*, defined as *t*, expressed as follows:

(2) $$\begin{array}{c} t\left(A⟶B\right)=\frac{\left(A\cup B\right).\text{con}}{n}. \end{array}$$

The incidence of *B* in transaction data containing *A* is called the credibility of association rules *A*⟶*B* and is represented by *d*, expressed as follows:

(3) $$\begin{array}{c} d\left(A⟶B\right)=\frac{\left(A\cup B\right).\text{con}}{A.\text{con}}. \end{array}$$

Firstly, all frequent item sets meeting the minimum support Minsup are obtained through frequent item set mining, and all items of the transaction set are searched to obtain frequent item set *Z*_*i*_ of different generations, until the non-empty candidate item set *D*_*i*_ cannot be generated. Then, strong association rules corresponding to frequent item sets are obtained through the association rule network mining method. The specific process of data mining based on the Apriori algorithm is shown in Figure 2.

In this study, the graphics processing unit (GPU) [20] was used for multi-threading parallel processing to optimize the traditional Apriori algorithm machine, so as to shorten the running time of the algorithm. For the support count of item *d* in the candidate item set *D*_*k*_, GPU is used to evenly distribute transaction database transactions to each thread, and item *d* is detected on each transaction set to obtain the respective count. Then, the support of the final candidate item set is calculated. The specific process of the Apriori algorithm medical big data mining after parallel optimization is shown in Figure 3.

### 2.3. The Terminal Design of the Cloud Follow-Up System

The cloud follow-up system mainly includes the log-in, my workstation, the patient records, follow-up center, satisfaction management, propaganda and education center, SMS platform, and appointment management module. The system log-in module mainly includes log-in, registration, and password retrieving. Each module includes the user name, password, and verification code information to validate input information. The specific content of the log-in module of the cloud follow-up system is shown in Figure 4.

My workstation module mainly includes my home page, my follow-up, health propaganda and education, and satisfaction survey. My home page mainly includes patient services, patient interventions, and hospital announcements. My follow-up mainly records patients' follow-up, appointment, and medical records. The health education is used to query the follow-up status of patients. The basic information such as patient name, age, gender, contact information, bed number, date of propaganda and education, ward environment introduction, and status of propaganda and education can be clearly displayed in the task list. The satisfaction survey part investigates the patient's nursing mode and the satisfaction of the cloud follow-up center. The details of my workstation module are shown in Figure 5.

The patient record module includes five parts of health profile, medical archives, business management, business records, and health monitoring. The health profile part displays the patient's personal information, hospitalization information, operation situation, outpatient examination, and physical examination information in detail. The medical archive part mainly includes hospital medical information and RCT information. Hospital medical information mainly concerns hospitalization information, operation time, operation name, surgeon, anesthesia method, operation level, incision healing level, anesthesiologist, examination report, and test report.  Figure 6 shows the specific content of patient record module of the cloud follow-up system.

The statistical central module mainly includes four parts: follow-up workload statistics, follow-up form statistics, health propaganda and education statistics, and satisfaction survey statistics.  Figure 7 shows the specific content of the statistical central module.

### 2.4. Server Design

Tomcat Server has the characteristics of stable operation, reliability, high efficiency [21], and good adaptability. It can work with most HTTP servers [22] and can run on Java Web application containers such as Servlet and Java Server Pages (JSP). Therefore, Tomcat is selected as the World Wide Web server in this study, and Servlet and JSP are mainly used as Java Web application containers. Servlet can respond to requests sent by the client in the form of text or pictures.  Figure 8 shows the server structure.

### 2.5. Database Design and Test Environment

MySQL database management system is characterized by small storage volume, fast query speed, and low development cost [23]. Database and its application system are the core of mobile intelligent medical system [24]. The design of database should meet the principles of integrity, less quantity, a smaller number of fields, and efficient operation [25]. The main physical structure of this database includes patient information table, nursing data table, nursing prescription table, and nursing data information table.  Table 1 presents the basic information of patients.  Table 2 shows the care information of patients.  Table 3 displays the care prescription of patients.  Table 4 presents patient care data.

The operating platform environment of the test system is as follows: computer operating system: Windows 10 Flagship 64 bit operating system, server-side scripting language: PHP 5.3.5, relational database management system: MySQL 5.5.8, Web server software: Apache 2.2.17, development environment: project development compiler Eclipse PHP Studio 3, data management library: MySQL, and code programming tools: JavaScript and Ajax.

### 2.6. Verification of Continuous Nursing Intelligent Medical System for Breast Cancer Patients after Surgery

The data for the verification are all from the postoperative follow-up database of breast cancer patients in the rehabilitation department of our hospital in the cloud follow-up intelligent medical system. The electronic medical record database records the complete diagnosis and treatment information of patients after breast cancer surgery, including the basic information of age, gender, and allergy history, treatment methods, postoperative nursing methods, patient nursing compliance, and the occurrence of complications. To protect patient privacy, the personal information was encrypted, and all researchers had signed a written agreement indicating that there was no attempt to gain access to the patient's private information. In this study, the case data of 379 patients from January 2019 to December 2020 were used, involving basic patient information, treatment methods, postoperative out-of-hospital nursing methods, and rehabilitation-related indicators. According to different nursing methods, the patients were divided into the control group (routine telephone follow-up) and the intervention group (continuous nursing intervention group), including 163 pieces of data in the control group and 216 pieces of data in the intervention group.

### 2.7. Statistical Methods

SPSS 19.0 statistical software was used for data processing. Mean ± standard deviation $\left(\bar{x}\pm S\right)$ was for measurement data, and the t-test was used. The count data were expressed as percentage (%), and *P* < 0.05 indicated statistically significant differences.

## 3. Result Analysis

### 3.1. The Relationship between Data Mining Running Time and Data Volume

Figure 9 shows the relationship between the running time of data mining process and the data volume. As the amount of data continues to increase, the running time of data mining shows an obvious upward trend; that is, there is a positive relationship between running time and data volume. When the amount of data is small (less than 400 items), the running time of data mining varies little under different amounts of data.

Figure 10 shows the relationship between data mining time and data volume under CPU and GPU. With the continuous increase in data volume, the running time of data mining shows an upward trend under both CPU and GPU, and the upward trend is more obvious under CPU. Under the same number of nodes, compared with CPU, the Apriori algorithm under GPU achieves an acceleration ratio of 6.67 times at large.

### 3.2. The Relationship between Running Time and the Number of Nodes

Figure 11 shows the running time of data mining under different data quantities and node numbers. With the increase in the node number, the running time gradually shows a downward trend. The reason is that the optimized Apriori algorithm can evenly distribute the data sets to nodes, and a higher number of nodes indicate a smaller amount of data processed by each node, thus significantly shortening the running time. At the same time, the amount of data processed by the Apriori after optimization also increases with the increase in the number of nodes, which is consistent with the above principle of average distribution of data. Therefore, the number of nodes in the cluster is inversely proportional to the running time of data mining.

### 3.3. Analysis of Nursing Compliance Based on the Intelligent Medical System

The intervention group and the control group were compared for the compliance of exercise behavior. The numbers of patients of complete compliance, partial compliance, poor compliance, and total compliance in the intervention group were 111 (68.10%), 45 (27.61%), 7 (4.29%), and 156 (95.71%), respectively. There were 110 patients (50.93%), 51 patients (23.61%), 55 patients (25.46%), and 161 patients (74.54%) in the control group, respectively, and there were statistical differences in the proportion of patients with complete compliance, the proportion of patients with poor compliance, and the proportion of total compliance (*P* < 0.05).  Figure 12 displays the comparison of compliance between the two groups.

### 3.4. Analysis of the Score of Quality of Life before and after Nursing Based on Intelligent Medical System

The quality-of-life scores of the two groups of patients before and after the nursing intervention were compared and analyzed. There was no significant difference in the quality-of-life scores between the two groups before the intervention (*P* > 0.05). After the intervention, the quality-of-life scores of the two groups were statistically different than those before (*P* < 0.05), and the *quality*-of-life score of the intervention group was higher than that of the control group after the intervention, and there was a statistical difference between the two (*P* < 0.05).  Figure 13 is the comparison of quality-of-life scores between the two groups before and after the intervention.

### 3.5. Analysis of Recovery Condition of the Affected Limb before and after Nursing Based on the Intelligent Medical System

A comparative analysis was made on the functional recovery degree of affected limbs in different time periods after the intervention between the intervention group and the control group. With the extension of intervention time, the number of affected limbs in the intervention group returning to the normal state increased significantly, and the proportion was significantly higher than that in the control group, and there was a statistical difference between the two groups (*P* < 0.05). The proportion of patients with limited and severely limited functional activity of the affected limb in the intervention group was significantly lower than that in the control group (*P* < 0.05).  Figure 14 is the comparison of functional recovery degree of affected limb between two groups.

### 3.6. Analysis of Postoperative Nursing Satisfaction Based on Intelligent Medical System

According to the statistical analysis of the total satisfaction of the two groups of patients with postoperative nursing based on the intelligent medical system, in the intervention group, 107 cases (65.64%), 44 cases (26.99%), and 12 cases (7.36%) were satisfied, basically satisfied, and dissatisfied, respectively, and there were 151 (92.64%) satisfied cases in total; in the control group, 67 cases (31.02%), 99 cases (45.83%), and 50 cases (23.15%) were satisfied, basically satisfied, and dissatisfied, and there were 166 (76.85%) satisfied cases in total. The satisfaction rate of postoperative nursing care in the intervention group was significantly higher than that in the control group, and there was a significant difference between them (*P* < 0.001). The proportion of patients who were basically satisfied with and dissatisfied with postoperative nursing in the control group was higher than that in the intervention group (*P* < 0.05). The total satisfaction of postoperative nursing in the intervention group was higher than that in the control group, and there was a statistical difference between them (*P* < 0.05).  Figure 15 shows the postoperative nursing total satisfaction analysis based on the intelligent medical system.

## 4. Discussion

The current research results show that the Apriori algorithm is the most time-consuming in the candidate item set support counting stage in the data mining process [26–28]. In this study, parallelization is adopted to accelerate the algorithm, and the results show that the running time of data mining is in positive proportion to the amount of data. When the amount of data is small, the running time of data mining varies little under different amounts of data. This is because the support process of the candidate item set after parallel optimization with a small amount of data takes a small amount of time in the whole program. With the increase in data amount, the time spent in the support counting process of the candidate item set takes a larger proportion in the running time, resulting in a significant extension of the running time [29]. When the amount of data is large, the counting time of the candidate set is proportional to the amount of data. The study shows that with the increase in data volume, the running time of data mining shows a rising trend under both CPU and GPU. Compared with CPU, the Apriori algorithm under GPU achieves a maximum acceleration ratio of 6.67 times. The reason is that the GPU parallel acceleration processing enables the nodes in the cluster to be configured into a security group, which improves the throughput [30] and then shortens the running time.

Exercise compliance mainly evaluates whether the exercise mode and duration of patients are consistent with the nursing plan formulated by medical staff [31]. The results showed that the proportion of patients with complete compliance, the proportion of patients with poor compliance, and the proportion of total compliance in the intervention group were statistically different (*P* < 0.05). It can be inferred that patients' compliance is higher under the continuous nursing mode based on mobile medical care, which is consistent with the research results of Lin et al. [32]. Under normal circumstances, the patients have psychological and physical problems during treatment, which have a serious impact on their quality of life after surgery. The relevant research results show that breast cancer patients have a high demand for health knowledge in the stable phase after surgery. Therefore, continuous nursing is needed for patients after surgery, which can maintain the treatment effect, prolong survival time, and improve the quality of life, playing an extremely important role after the surgery [33]. The results of this study showed that after the intervention, the quality-of-life scores of patients in the two groups were statistically different from those before the treatment (*P* < 0.05), and the quality-of-life scores of patients in the intervention group were higher than those in the control group (*P* < 0.05). This indicates that continuous nursing intervention can effectively help patients improve their quality of life. The traditional nursing model for breast cancer patients after surgery was only the simple guidance before discharge and oral education during reviews, which was affected by many factors such as time, space, financial resources, and manpower. As a result, the nursing effect achieved was often not satisfactory [34]. With the application of the intelligent medical system, the continuous nursing benefits breast cancer patients a lot in terms of costs and hospital stay [35]. It has gradually replaced the traditional nursing model and is widely recognized by the whole society. The study showed that the satisfaction rate of postoperative nursing in the intervention group was significantly higher than that in the control group (*P* < 0.001), and the proportion of basically satisfied and dissatisfied patients in the control group was higher than that in the intervention group (*P* < 0.05). The total satisfaction of postoperative nursing in the intervention group was higher than that in the control group (*P* < 0.05) [36, 37]. After the intervention, the proportion of the patients with the affected limb function returning to normal in the intervention group was significantly higher than that in the control group (*P* < 0.05), and the proportion of patients with limited and severely limited functional activity of the affected limb in the intervention group was significantly lower than that in the control group (*P* < 0.05) [38, 39]. It suggests that it is necessary to implement cloud-based continuous nursing intervention for patients after breast cancer surgery, and it can be widely promoted in the clinic as a routine nursing mode for such patients in the future, so that more patients can benefit from it and obtain more ideal outcomes and prognoses [40–42].

## 5. Conclusion

In this study, the Apriori algorithm is introduced to optimize the mining technology of big data. Then, the intelligent mobile medical communication system is established to evaluate the intervention effect of different nursing methods on patients undergoing breast cancer surgery. It shows that the intelligent mobile medical communication system established in this study can effectively evaluate the intervention effect of different nursing methods on patients undergoing breast cancer surgery. However, there are still some shortcomings in this study. This study only analyzes the compliance, the satisfaction degree, and the mobility function of affected limbs of breast cancer patients. There is no further analysis of patients' complications. In the future, relevant questionnaires will be designed to further investigate patients' complications, and the results will be applied to out-of-hospital continuing nursing of other diseases to expand the application scope. In conclusion, the intelligent mobile medical communication system established in this study has potential application value, which provides a new idea for the evaluation of postoperative intervention effect under big data.

## Figures and Tables

**Figure 1:** Overall framework of intelligent follow-up medical system based on the cloud platform.

**Figure 2:** Data mining flowchart of the Apriori algorithm.

**Figure 3:** Flowchart of big data mining with the optimized Apriori algorithm.

**Figure 4:** The log-in module of the cloud follow-up system.

**Figure 5:** My workstation module of the cloud follow-up system.

**Figure 6:** Patient record module of the cloud follow-up system.

**Figure 7:** Statistical central module of the cloud follow-up system.

**Figure 8:** Server architecture diagram.

**Figure 9:** Relationship between data mining running time and data volume.

**Figure 10:** Relationship between data mining running time and data volume under different conditions.

**Figure 11:** Relationship between running time and number of nodes.

**Figure 12:** Comparison of compliance between the two groups (^*∗*^represents a statistical difference compared with the control group, *P* < 0.05).

**Figure 13:** Comparison of quality-of-life scores between the two groups before and after the intervention (^*∗*^ represents statistical differences compared with before intervention, *P* < 0.05; # represents statistical differences compared with the control group, *P* < 0.05).

**Figure 14:** Comparison of functional recovery degree of affected limb between two groups (^*∗*^ represents a statistical difference compared with the control group, *P* < 0.05).

**Figure 15:** Postoperative nursing total satisfaction analysis based on the intelligent medical system (^*∗*^ represents a statistical difference compared with the control group, *P* < 0.05; ^*∗∗*^ shows significant differences compared with the control group, *P* < 0.01; and ^*∗∗∗*^ represents a significant difference compared with the control group, *P* < 0.001).

**Table 1:** Basic information of patients.

Field name	Data type	Type or not	Length	Remark
ID code	int	Yes	20	Not null
Name	tinyint	No	5	Not null
Sex	varchar	No	2	Not null
Age	datetime	No	0	Not null
Marriage	varchar	No	10	Null
Profession	varchar	No	10	Not null
Educational background	varchar	No	10	Not null

**Table 2:** Care information of patients.

Field name	Data type	Type or not	Length	Remark
ID code	int	Yes	20	Not null
History of diseases	varchar	No	400	Not null
Obstetrical history	datetime	No	50	Not null
Diagnostic time	Year	No	4	Not null
Diagnostic result	varchar	No	200	Not null
Nursing method	varchar	No	400	Not null
Nursing goal	int	No	120	Null
Nursing plan	varchar	No	40	Null

**Table 3:** Care prescription of patients.

Field name	Data type	Type or not	Length	Remark
ID code	int	No	20	Not null
Doctor ID	int	No	20	Not null
Time to start nursing	datetime	Yes	0	Not null
Nursing prescription	varchar	No	500	Not null

**Table 4:** Patient care data.

Field name	Data type	Type or not	Length	Remark
ID code	int	Yes	20	Not null
Data type	int	No	11	Not null
Data name	varchar	No	50	Not null
Data content	Mediumblob	No	0	Not null
Score	int	No	5	Not null

## Data Availability

The simulation experimental data used to support the findings of this study are available from the corresponding author upon request.
